# VVC In-Loop Filtering Based on Deep Convolutional Neural Network

**DOI:** 10.1155/2021/9912839

**Published:** 2021-07-07

**Authors:** Soulef Bouaafia, Seifeddine Messaoud, Randa Khemiri, Fatma Elzahra Sayadi

**Affiliations:** ^1^University of Monastir, Laboratory of Electronics and Microelectronics, Faculty of Sciences of Monastir, Monastir, Tunisia; ^2^University of Gabes, Higher Institute of Computer Science and Multimedia of Gabes, Gabes, Tunisia; ^3^University of Sousse, National Engineering School of Sousse, Sousse, Tunisia

## Abstract

With the rapid advancement in many multimedia applications, such as video gaming, computer vision applications, and video streaming and surveillance, video quality remains an open challenge. Despite the existence of the standardized video quality as well as high definition (HD) and ultrahigh definition (UHD), enhancing the quality for the video compression standard will improve the video streaming resolution and satisfy end user's quality of service (QoS). Versatile video coding (VVC) is the latest video coding standard that achieves significant coding efficiency. VVC will help spread high-quality video services and emerging applications, such as high dynamic range (HDR), high frame rate (HFR), and omnidirectional 360-degree multimedia compared to its predecessor high efficiency video coding (HEVC). Given its valuable results, the emerging field of deep learning is attracting the attention of scientists and prompts them to solve many contributions. In this study, we investigate the deep learning efficiency to the new VVC standard in order to improve video quality. However, in this work, we propose a wide-activated squeeze-and-excitation deep convolutional neural network (WSE-DCNN) technique-based video quality enhancement for VVC. Thus, the VVC conventional in-loop filtering will be replaced by the suggested WSE-DCNN technique that is expected to eliminate the compression artifacts in order to improve visual quality. Numerical results demonstrate the efficacy of the proposed model achieving approximately −2.85%, −8.89%, and −10.05% BD-rate reduction of the luma (*Y*) and both chroma (*U*, *V*) components, respectively, under random access profile.

## 1. Introduction

With emerging technologies that have rapidly evolved, multimedia services and video applications have significantly increased. Therefore, higher resolution (4K and 8K), especially for video games, e-learning, video conferencing, and surveillance tasks, is required to meet end-users viewing quality specifications. A next generation video encoding, established by the Joint Video Experts Team (JVET) in July 2020 [1], was the successor of high efficiency video coding (HEVC) [2]; it is the versatile video coding (VVC), which was also called H.266. VVC achieves a BD-rate savings up to 30% at the same quality as HEVC, which is the best standard adopted to offer an appropriate level of performance for new multimedia services. Although VVC aims to keep high-quality compressed video with additional encoding features, it still inevitably suffers from compression artifacts, which can lead to a decrease in the video quality. Therefore, VVC's quality compressed video and images need to be improved. In this case, loop filters play a crucial role in video and image quality optimization before they are used for interprediction as reference images.

In the same way, as for HEVC, in order to remove video compression artifacts and improve reconstructed video quality, VVC standard adopts the loop filtering technique, including the deblocking filter (DBF), sample adaptive offset (SAO), and adaptive loop filter (ALF). The DBF is designed to eliminate artifacts along block borders using discontinuity-based smoothing filters [3, 4]. Then, SAO is the second filter applied after DBF in HEVC and VVC [5], for compensating the reconstructed samples with different offset values in order to remove ringing effects.

ALF is a modern VVC function that removes distortions between restored and original images that are the most current loop filters [6]. Although traditional in-loop filters can alleviate those artifacts, the dynamic distortion produced by video compression is hard to resolve. Deep learning progress is known to be a strong technology to overcome this task, by using the convolutional neural network (CNN) as the most versatile and effective computational method for images and videos detection and analysis [7].

In order to increase the video quality, many CNN filtering methods have been suggested for HEVC and VVC standards [8–12]. These existing methods are proposed to minimize visual artifacts and to achieve great efficiency through CNN-based in-loop filtering and postprocessing. For example, Jia et al. in [8] proposed a HEVC postprocessing residue-guided loop filter. A deep network based on progressive rethinking and collaborative learning mechanisms was developed by Wang et al. in [9] to enhance the quality of the reconstructed frame for intra and interprediction. Inspired by emerging technology challenges, as well as high speed rate and high video and image resolution quality, the original in-loop filtering has become inadequate to satisfy the services demanded by the end users. In this study, we propose a powerful deep CNN-based filtering technique, called the wide-activated squeeze-and-excitation deep convolutional neural network (WSE-DCNN). The proposed technique provides powerful new loop filtering using typical VVC standards (DBF, SAO, and ALF). The goal is to effectively eliminate compression artifacts and improve the reconstructed video quality and then meet the end-users services. The purpose of this article is to propose a WSE-DCNN technique-based quality enhancement and then to implement the scheme proposed in the VVC standard, which provides coding gains accordingly for the random access configuration.

The remainder of this study is organized as follows: Section 2 presents the related work overview. The proposed deep CNN-based in-loop filtering for VVC standard is defined in Section 3. Then, in Section 4, the proposed method is evaluated. Finally, Section 5 concludes the study.

## 2. Related Work Overview

In recent years, artificial intelligence has seen tremendous progress in computer vision topics, in particular in image and video compression [13–15]. Deep learning networks have been applied to enhance coding tools for HEVC and VVC standards, including intra and interprediction, transformation, quantization, and loop filtering [16, 17]. With regards to the HEVC, Bouaafia et al. in [14] proposed a reduction of HEVC complexity based on machine learning in the process of interprediction, which saves a good performance in terms of RD cost and computational complexity. Furthermore, a fast CNN-based algorithm is developed by Yeh et al. in [18] to improve the efficiency of HEVC intracoding. Pan et al. in [19] suggested an improved ED-CNN-based in-loop filtering to replace HEVC DBF and SAO in order to remove artifacts. The results prove that the proposed algorithm achieves BD-rate savings of 6.45% and PSNR gains of 0.238 dB. A novel technique for DBF and SAO in HEVC intracoding was proposed based on the Variable-filter-size Residue learning convolutional neural network (VRCNN) [20]. The obtained results show that the suggested technique achieves 4.6% BD-rate savings.

In order to enhance loop filtering and postprocessing, Ma et al. in [10] have developed a new CNN model, known as MFRNet for the VVC standard. The proposed model was implemented into the VVC test model to alleviate visual errors and increase video quality. In addition, a dense residual convolutional neural network (DRN) for the VVC filtering method proposed was applied after DBF and before SAO and ALF [12]. The H.265/VVC fast-intra-CU coding technique is based on the improved DAG-SVM classifier to minimize CU partition complexity [21]. Achieved results reveal that the proposed method achieves a 54.74% time saving. Moreover, Park et al. in [22] proposed to use a lightweight neural network (LNN) for the fast decision algorithm to remove redundant VVC block partitioning.

The suggested model provides a compromise between the compression and encoding complexity. In this study, we propose a wide-activated squeeze-and-excitation deep CNN- (WSE-DCNN-) based in-loop filtering approach for VVC video quality enhancement and achieve coding gains.

## 3. Proposed Method

### 3.1. Proposed WSE-DCNN-Based In-Loop Filtering for VVC

The VVC standard [1] still employs the block-based hybrid video coding architecture used in all video compression standards, since H. 261. It includes intraframe prediction, interframe prediction, transformation, quantization, loop filtering (DBF, SAO, and ALF), and entropy coding.  Figure 1 depicts the block diagram of a hybrid video encoder. The VVC architecture is made up of two processes, such as encoder and decoder processing. Each picture is split into block-shaped regions, with the exact block partitioning, called coding tree unit (CTU), which is the basic block partition of the HEVC and VVC standards. The first picture of a video sequence is coded using only intrapicture prediction. For all remaining pictures of a sequence or between random access points, interpicture temporally predictive coding modes are typically used for most blocks. The encoding process for interpicture prediction consists of choosing motion data comprising, the selected reference picture, and motion vector to be applied for predicting the samples of each block. The residual signal of the intra or interpicture prediction, which is the difference between the original block and its prediction, is transformed by a linear spatial transform. The transform coefficients are then scaled, quantized, entropy-coded, and transmitted together with the prediction information. The encoder duplicates the decoder processing loop, such that both will generate identical predictions for subsequent data. Therefore, the quantized transform coefficients are constructed by inverse scaling and are then inverse transformed to duplicate the decoded approximation of the residual signal. The residual is then added to the prediction, and the result of that addition may then be fed into the loop filters (including, DBF, SAO, and ALF) to smooth out artifacts induced by block-wise processing and quantization. The final picture representation (the output of the decoder) is stored in a decoded picture buffer to be used for the prediction of subsequent pictures.

In our study, the proposed WSE-CNN model replaces the original VVC loop filtering module (including, DBF, SAO, and ALF), as shown in Figure 1. The principal goal of this strategy is to improve the visual quality of the reconstructed frame while maintaining coding gains. The rate distortion optimization (RDO) technique is used to determine whether to apply to each coding unit (CU) the proposed WSE-DCNN in-loop filter. Equation (1) is given for the RDO metric.

(1) $$\begin{array}{c} J=D+\lambda R, \end{array}$$

where the distortion between the original and the reconstructed frame is denoted by *D*, the coding bits needed represents by *R* and the Lagrange multiplier controlling the trade-off between *D* and *R* is *λ*. The coding tree unit (CTU) level on/off control is adopted to avoid a reduction in RDO performance. The frame-level filtering would be shut off to prevent oversignal, if the enhancement quality is not worth to cost the signaled bits. Specifically, the control flags at the CTU-level and frame-level are designed as follows. For each CTU, if the RD performance of the filtered CTU achieves better quality, the corresponding CTU control flag is enabled; otherwise, the flag is disabled. After all the CTUs in one frame are determined, the frame-level RD cost before and after filtering are calculated in equation (1) indicated by *J*1 and *J*2, respectively. If *J*1 > *J*2, the frame-level flag will be enabled. Hence, the corresponding frame-level flag can be encoded in the slice header and CTU-level control flags can be signaled into each corresponding CTU syntax. Otherwise, the frame-level flag is disabled and CTU-level flags will not be encoded for transmission anymore.

### 3.2. WSE-DCNN Architecture

Figure 2 shows the proposed framework. The suggested technique, divided into two chromas (*U* and *V*) and luma (*Y*), would filter out the three components simultaneously. The WSE-DCNN model proposed consists of six inputs; three are YUV reconstructed and the other three include the QP quantization parameter and the luma and chroma coding unit. These inputs are first normalized to provide better convergence in the training process and then fed to the proposed model. Hence, the three (*Y*/*U*/*V*) reconstructions are normalized to [0, 1] based on the highest bit depth value. This means that the normalized values (*P*′(*x*, *y*)) are achieved by the following equation.

(2) $$\begin{array}{c} P^{\prime \prime }\left(x,y\right)=\frac{P\prime \left(x,y\right)}{1\ll B-1},\;x=1,\ldots ,W,\;y=1,\ldots ,H, \end{array}$$

where *B* denotes the bit depth, *P*^″^(*x*, *y*) is the normalized value in normalized *Y*/*U*/*V* at (x,y), and *W* and *H* are the width and the height of the reconstructed frame, respectively.

Various quantization parameters (QPs) contribute to a variety of reconstructed video quality. This makes it easier to use a single set of parameters to fit reconstructions with different qualities. QP should be normalized to QPmap (3).

(3) $$\begin{array}{c} \text{QPmap}\left(x,y\right)=\frac{\text{QP}}{63},\;x=1,\ldots ,W,\;y=1,\ldots ,H. \end{array}$$

The CU partition of the luma (*Y*) and chroma (*U*,  *V*) components also represents the inputs. Since the blocking artifacts are mainly caused by CU block partition, the division information of CU is converted into coding unit maps (CUmaps) and normalized. For example, for each CU in each frame, the boundary position is filled with two and the other positions are filled with one. However, the normalization factor is two, and two CUmaps can be obtained, one as *Y* − CUmap and the other denoted by UV − CUmap.

The WSE-DCNN process has three levels, as shown in Figure 2. The three *Y*,  *U*,  *V* components are processed via WSE blocks at the first level, and each component is fused with its own CUmap. Moreover, before it is concatenated to feature maps, CUmap would be multiplied by its own channel. Since *U*' and *V*' size is just the half of *Y*, the above needs to be used for size alignment. In the second level, the feature maps of different channels are connected together and then processed by several WSE blocks. At this level, the QPmap is also concatenated. At the last level, in order to produce the output residual image, the three channels are processed separately again.The WSE is the principal module for the proposed WSE-DCNN-based in-loop filtering technique, as shown in Figure 3. Furthermore, the wide-activated convolution [23] and the squeeze-and-excitation (SE) operation [24] compose this simple module. The wide-activated convolution performs very well in super-resolution and noise reduction tasks. It composed of 3 × 3 wide convolution followed by the rectified linear unit (ReLU) [25] activation function and a convolution layer with kernel size 1 × 1. Next comes the SE operation, the most used operation to weigh each convolutional layer. It can use the complex relationship between different channels and generate a weighting factor for each channel.

The WSE module includes the following steps as shown in Figure 3, given a feature map *X* with shape *H* × *W* × *C*, where *C* means the channel amounts. First, given *Y*_1_ and *Y*_2_ are the outputs of the wide-activated convolution, as shown in the following equations.

(4) $$\begin{array}{c} Y_{1}=\text{ReLU}\left(W_{1}X+b_{1}\right), \end{array}$$

(5) $$\begin{array}{c} Y_{2}=W_{2}Y_{1}+b_{2}. \end{array}$$

In the second step, each channel obtains a value according to the squeeze operation using global average pooling (GAP) *Y*_3_(*k*).

(6) $$\begin{array}{c} Y_{3}\left(k\right)=\frac{1}{\text{H}\times \text{W}}\sum_{i=1}^{H}\sum_{j=1}^{W}Y_{2}\left(i,j,k\right). \end{array}$$

The excitation operation is described by two fully connected layers followed by ReLU and sigmoid (*σ*) activation functions, respectively. *Y*_4_ is the first fully connected layer followed by ReLU, which is refined by a certain ratio *r*. Then, the second fully connected layer followed by the sigmoid activation function is denoted by *Y*_5_, and it gives each channel a smoothing gating ratio in the range of [0, 1].

(7) $$\begin{array}{c} Y_{4}=\text{ReLU}\left(W_{4}Y_{3}+b_{4}\right),\\ Y_{5}=\sigma \left(W_{5}Y_{4}+b_{5}\right). \end{array}$$

According to the WSE function, each *Y*_2_ channel is multiplied by the gating ratio.

(8) $$\begin{array}{c} Y_{6}\left(i,j,k\right)=Y_{2}\left(i,j,k\right)\times Y_{5}\left(k\right)\\ \forall i\in \left\{1,\ldots ,H\right\},\forall j\in \left\{1,\ldots ,W\right\},\forall k\in \left\{1,\ldots ,C\right\}. \end{array}$$

Finally, when the number of input equals to the output channels *C*, a skip connection will be added directly from input to output to learn the residue. Otherwise, there is no skipped connection.

## 4. Results and Discussion

The efficiency of the proposed WSE-DCNN-based in-loop filtering scheme under VVC standards is assessed in this section. Then, a comparative performance with the existing approaches is introduced.

### 4.1. Training Settings

In this contribution, the public video dataset (BVI-DVC) is exploited to train the deep video compression techniques [26]. The BVI-DVC dataset contains 800 video sequences with different resolutions between 270p and 2160p. In this case, we choose 80% video sequences for the training process and 20% for the validation phase. These sequences are compressed under random access scenario by the VVC VTM-4.0 test model [27] with QP values (22, 27, 32, and 37). For each QP, the reconstruction video images, including luma and chroma components, and its corresponding ground truth are divided into 64×64 patches, which were selected in a random order.

The proposed deep learning framework is trained offline in a supervised learning manner. The deep framework used during the training phase is the TensorFlow-GPU [28]. In the experiments, the training parameters used are denoted by the following: the batch size is set to 128, the training epochs to 200, the learning rate is set to 0.001, and weight decay of 0.1 for every 50 epochs. To train the proposed deep model, we applied an optimizer, such as the Adam algorithm [29]. Intel®core TM i7-3770 @3.4 GHz CPU with 16 GB RAM and an NVIDIA GeForce RTX 2070 GPU are used as the training platforms.

To train the proposed WSE-DCNN model, we assume that the mean square error (MSE) [30] is applied as the loss function between the reconstructed and the ground truth image. The MSE loss function is defined in the following equation.

(9) $$\begin{array}{c} L\left(\theta \right)=\frac{1}{N}\sum_{i=1}^{N}{\left\|F\left(Y_{i},\theta \right)-X_{i}\right\|}_{2}^{2}, \end{array}$$

Let *X*_*i*_ is the ground truth of the proposed model, where *i* ∈ {1,…, *N*}. F(.) is the output of the WSE-DCNN model, where *Y*_*i*_ represents the compressed images, *i* ∈ {1,…, *N*}, and *θ* is the parameter set of the proposed framework.

The loss function evaluation is the way to judge whether the model is well trained or not. It indicates, as shown in Figure 4, that the model converged reasonably quickly by tending to zero the loss function. In addition, the loss (defined in equation (9)) value remains the same from epoch 100 onwards, which means that no training problem arose during the training process. This proves that model's weight is well tuned.

The proposed WSE-DCNN technique is implemented in the VVC standard in order to replace the conventionally applied filtering system during the testing process. All experiments are evaluated using a random access configuration at four QP values (22, 27, 32, and 37) under the VVC JVET common test conditions (CTC) [31]. The RD performance analysis is performed based on Bjøntegaard-delta bitrate (BD-rate) [32]. The BD-rate represents the average bitrate saving calculated between two RD curves for the same video quality, where negative BD-rate values indicate actual bitrate saving and positive values indicate how much the bitrate is increased.

### 4.2. RD Performance Evaluation

Compared to the original VVC standard, Table 1 provides the RD performance results of the proposed technique. Columns *Y*, *U*, and *V* in the table show the BD-rate of *Y*, *U*, and *V* components, respectively.

The proposed technique achieves better mean coding gains when integrated into VVC standard. It can achieve 2.85% BD-rate savings for luma *Y* component and 8.89% and 10.05% for both chroma *U* and *V* components under random access profile, as given in Table 1. The proposed system provides substantial efficiency of RD compression primarily for all test sequences in *U* and *V* chrominance. It is also apparent that, for some sequences, the compression performance varies widely, such that video sequence content affects the proposed model. In addition, the suggested model performs better in terms of RD performance for high motion or rich texture video sequences, such as Campfire, CatRobot1, Kimono2, RaceHorses, and BQSquare. Consequently, the suggested CNN-based loop filtering outperforms VVC with the conventional loop filtering algorithm in terms of RD performance.

PSNR is also used as a quality metric to test the performance of our proposed filtering technique integrated into the VVC standard, which is defined by the following equation [33].

(10) $$\begin{array}{c} {\text{PSNR}}_{\text{YUV}}=\frac{6\times {\text{PSNR}}_{Y}+{\text{PSNR}}_{U}+{\text{PSNR}}_{V}}{8}. \end{array}$$

In order to show the subjective visual quality and to further verify the effectiveness of the suggested model, the RaceHorses video sequence for class D was encoded by QP 22 under random access profile.  Figure 5 shows the visual quality comparison. It is obvious that frame details are blurry when compressed by the original VVC standard, but become clearer after being filtered by the proposed technique. In contrast to the regular VVC with/without conventional in-loop filtering, the proposed technique effectively removes all blocking artifact, such as ringing and blurring artifacts, which enhances video quality.

A comparative performance of the proposed approach was made with other CNN-based filtering methods, as given in Table 2. Based on VVC CTC, Table 2 provides the comparison of the encoding performance in terms of reducing RD performance with other approaches [12, 33]. In this work [12], Chen et al. proposed to improve reconstructed video quality through the in-loop filter of a dense residual convolutional neural network (DRN). This network is placed after DF and before SAO and ALF into VVC VTM-4.0 reference software, in which the DIV2K dataset [34] is used in the training phase. In addition, for both inter and intraimages, the CNN in-loop filter algorithm is proposed [33], which is implemented in VVC VTM-4.0 before ALFs with DBF and SAO are disabled.

Compared to other previous approaches, for all test sequences from class A1 to class D, the proposed WSE-DCNN system implemented in VVC better performed in terms of compression performance for both luma and chroma components, as given in Table 2. This means that in terms of objective and subjective visual quality, the model proposed works well. As results of the proposed technique, the effectiveness of the WSE-DCNN approach is shown in comparison to other approaches in almost all test sequences.

We presented a RD performance curves for the suggested model-based in-loop filtering, compared to other approaches with QPs values under random access scenario for class A1 to class D. The RD performance curves comparisons are given in Figure 6. Comparing the corresponding methods, we can see that the proposed filter model considerably enhances the VVC compression performance. The in-loop filtering suggested works well, in particular, in high-resolution video sequences, such as in class A1, class A2, and class B.

## 5. Conclusion

In this article, we have introduced a deep learning technique to improve VVC video quality while enhancing the user's services. To alleviate the coding artifacts as well as ringing, blocking, and blurring, the proposed WSE-DCNN technique is integrated into VVC standard to replace the traditional in-loop filtering. Compared to original VVC filters, simulation results show that the proposed system offers best objective and subjective compression efficiency, with a BD-rate reduction of approximately −2.85%, −8.89%, and −10.05% for *Y*, *U*, and *V* components, respectively. The comparative results reveal that the proposed in-loop filtering framework proves its effectiveness in improving video quality. In future work, two deep learning algorithms will be developed, one to improve the VVC CU partition at interprediction in order to reduce VVC complexity reduction and the other to replace original filters to enhance visual quality.

## Figures and Tables

**Figure 1:** Proposed WSE-DCNN-based in-loop filtering in VVC standard.

**Figure 2:** WSE-DCNN structure.

**Figure 3:** WSE module.

**Figure 4:** Training analysis “Loss curve.”

**Figure 5:** Visual quality comparison (the 26^th^ frame of RaceHorses with QP = 22: (a) Original; (b) VVC without in-loop filtering (PSNR=39.84 dB); (c) VVC (PSNR=39.96 dB); (d) VVC-based proposed model (PSNR=40.15 dB).

**Figure 6:** Comparative RD performance curves. (a) Class A1 “Campfire @ 3840 × 2160.” (b) Class A2 “CatRobot @ 3840 × 2160.” (c) Class B “BasketballDrive @ 1920 × 1080.” (d) Class C “BasketballDrill @ 832 × 480.” (e) Class D “BasketballPass @ 416 × 240.”

**Table 1:** VVC performance evaluation of the proposed model under random access profile.

Class	Sequences	BD-rate (%)		
		*Y*	*U*	*V*
Class A1	Tango2	−2.89	−10.02	−11.35
	Campfire	−1.22	−2.75	−10.28

Class A2	CatRobot1	−1.89	−10.76	−8.03
	DaylightRoad2	−1.47	−12.36	−2.55

Class B	Kimono2	−0.51	−8.13	−20.63
	ParkScene	−4.18	−9.25	−12.94
	Cactus	−2.36	−12.27	−9.70
	BasketballDrive	−2.53	−4.83	−7.82
	BQTerrace	0.11	−2.88	0.63

Class C	BasketballDrill	−3.84	−7.01	−9.97
	BQMall	−3.89	−11.48	−10.92
	PartyScene	−4.65	−9.69	−9.63
	RaceHorses	−1.35	−10.70	−13.66

Class D	BasketballPass	−3.40	−8.21	−7.79
	BQSquare	−5.27	−4.39	−11.44
	BlowingBubbles	−4.15	−8.52	−5.19
	RaceHorses	−5.08	−18.04	−19.74

**Overall**		**−2.85**	**−8.89**	**−10.05**

**Table 2:** Comparative RD performance with other approaches.

Class	Approach [12]			Approach [33]			Proposed approach		
BD-rate (%)	*Y*	*U*	*V*	*Y*	*U*	*V*	*Y*	*U*	*V*
Class A1	−1.27	−3.38	−5.10	0.87	0.12	0.22	−2.05	−6.38	−10.81
Class A2	−2.21	−5.74	−2.88	−1.12	−0.52	−2.11	−1.68	−11.56	−5.29
Class B	−1.13	−4.73	−4.55	−0.83	−0.47	−1.20	−1.89	−7.47	−10.09
Class C	−1.39	−3.63	−4.36	−1.76	−3.64	−6.80	−3.43	−9.72	−11.05
Class D	−1.39	−1.96	−3.08	−2.95	−3.27	−7.35	−4.47	−9.79	−11.04
**Overall**	−1.47	−3.88	−3.99	−1.16	−1.56	−3.44	**−2.70**	**−8.98**	**−9.65**

## Data Availability

The data used to support the findings of this study are available from the corresponding author upon request.
